# Comprehensive Characterization of Common and Cancer-Specific Differently Expressed lncRNAs in Urologic Cancers

**DOI:** 10.1155/2021/5515218

**Published:** 2021-07-09

**Authors:** You-Ji Yan, Ling Zhang, Jia-Jie Zhou, Zhong-Jun Chen, Yi-Xiang Liao, Jin-Min Zeng, Hao Shen

**Affiliations:** ^1^Department of Urology, Jingzhou Central Hospital, The Second Clinical College, Yangtze University, Jingzhou, Hubei 434020, China; ^2^Department of Pathology, Wuhan No. 1 Hospital, Tongji Medical College, Huazhong University of Science and Technology, Wuhan, Hubei Province 430022, China; ^3^Department of Urology, The Central Hospital of Wuhan, Tongji Medical College, Huazhong University of Science and Technology, Wuhan, Hubei Province 430014, China

## Abstract

Urologic cancers, comprising prostate carcinoma (PCa), renal cell carcinoma (RCC), and bladder carcinoma (BCa), were the commonly occurred carcinoma amid males. Long noncoding RNAs (lncRNAs) with the length of more than 200 nt functioned importantly in physiological and pathological advancement. Nevertheless, further investigation regarding lncRNA expression feature and function in urologic cancers should be essential. This study is aimed at uncovering the roles of the differently expressed lncRNAs in urologic cancers. The data of gene expression levels was downloaded from lncRNAtor datasets. The lncRNA expression pattern existing in different urologic cancers was assessed by hierarchical clustering analysis. Gene Ontology (GO) analysis and KEGG pathway analysis were separately applied to evaluate the biological function and process and the biological pathways involving differently expressed lncRNAs. Our results indicated that 18 lncRNA expressions were increased, and 16 lncRNA expressions were reduced in urologic cancers after comparison with that in normal tissues. Moreover, our results demonstrated 61, 422, 137, and 281 lncRNAs were specifically dysregulated in bladder cancer (BLCA), kidney renal clear cell cancer (KIRC), kidney renal papillary cell cancer (KIRP), and prostate adenocarcinoma (PRAD), respectively. Bioinformatics analysis showed that differently expressed lncRNAs displayed crucially in urologic cancers. The prognostic value of common and cancer-specific differently expressed lncRNAs, such as PVT1, in cancer outcomes, was emphasized here. Our research has deeply unearthed the mechanism of differently expressed lncRNAs in urologic cancers development.

## 1. Introduction

The data of human genome sequencing revealed most of RNA transcripts deriving from nonprotein-coding were transcribed from more than 90% of the human genome [1]. Long noncoding RNAs (lncRNAs) with the length of more than 200 nt functioned importantly in the tumorigenesis and progression with the increasing reports [2]. Previous studies revealed lncRNA expression was altered in multiple human carcinomas, such as breast carcinoma, liver carcinoma, lung carcinoma, and gastric carcinoma. lncRNAs could promote carcinoma progression. For instance, lncRNA YIYA induced glycolysis in breast cancer [3]. Meanwhile, lncRNAs could also suppress cancer progression, for example, lncRNA OCC-1 hindered colorectal cancer cell growth [4]. lncRNAs played their roles by epigenetically, transcriptionally, posttranscriptionally, and translationally regulating targets and participated in a large number of biological processes modulation, containing cell growth, metastasis, and apoptosis. For instance, The PVT1 lncRNA is a novel epigenetic enhancer of MYC and a promising risk-stratification biomarker in colorectal cancer [5]. PVT1 promotes gemcitabine resistance of pancreatic cancer via activating Wnt/*β*-catenin and autophagy pathway through modulating the miR-619-5p/Pygo2 and miR-619-5p/ATG14 axes [6]. PVT1 upregulation is a poor prognosticator and serves as a therapeutic target in esophageal adenocarcinoma [7]. In prostate cancer, PVT1 signals an androgen-dependent transcriptional repression program in prostate cancer cells and a set of the repressed genes predicts high-risk tumors [8]. Nevertheless, the function of most lncRNAs among cancers was not well understood.

Urologic cancers contained prostate carcinoma (PCa), renal cell carcinoma (RCC), and bladder carcinoma (BCa). In 2008, there were approximately 1,607,602 newly diagnosed urologic cancer cases worldwide, accounting for almost a quarter of the total number of human cancers [9, 10]. Bladder cancer (Bca) was ranked fourth among malignant tumors in males in the United States and eighth in the number of deaths. Prostate cancer is the most common type of cancers in male [11], Kidney cancer could be divided into different subtypes according to its different morphological and histological characteristics and genomic characteristics including renal clear cell carcinoma, papillary cell carcinoma, chromophobe renal cell carcinoma, collecting duct carcinoma, MiT family Translocation renal cell carcinoma, mucinous tubular and spindle cell carcinoma, and unclassified renal cell carcinoma [12]. Among these types, kidney renal clear cell cancer (KIRC) is the most common pathological type of RCC, accounting for more than 70% of kidney malignancies. KIRP is the second most common pathological type of RCC, accounting for about 15% of kidney malignancies. Some lncRNAs were reported to participate in urologic cancer prognosis and development. For instance, the androgen receptor-regulated prostate cancer progression was promoted by lncRNA ARLNC1 [13]. Xiao et al. found that energy metabolism mediated by c-Myc and tumor progression of renal could be inhibited by FILNC1 produced by energy stress [14]. lncRNA BLACAT2 was reported to promote bladder cancer-associated lymphatic metastasis [15]. There is a correlation existing in SNP polymorphism of H19 and decreases the risk of BCa [16]. However, a systematic understanding of common and cancer-specific lncRNAs of the function of urologic cancers was insufficient.

We for the first time identified common and cancer-specific differently expressed lncRNAs in urologic cancers here. Then, the coexpression network and GO along with KEGG analyses were individually applied to survey differently expressed lncRNA roles in urologic cancers. Our results suggested that lncRNAs functioned importantly in the modulation of the progression of urologic cancers, implying that it was a probable prospective biomarker at the molecular level.

## 2. Materials and Methods

### 2.1. Microarray Datasets and Data Preprocessing

Here, the expression levels of genes in kidney renal clear cell carcinoma (KIRC), kidney renal papillary cell carcinoma (KIRP), and prostate adenocarcinoma (PRAD) were downloaded from lncRNAtor datasets (http://lncrnator.ewha.ac.kr/index.htm) [17]. The differently expressed gene expression existing in normal and cancer samples was defined as the ∣ fold change (FC)  |  thresholds > 1.5 and *P* < 0.001.

### 2.2. Hierarchical Clustering Analysis

The lncRNA expression pattern amid different urologic cancers was assessed by the hierarchical clustering analysis. Cluster and TreeView programs were applied to conduct an analysis of the most significant differently expressed lncRNAs.

### 2.3. Gene Ontology (GO) and KEGG Pathway Analyses

The extract and analysis of biological molecule relationships from the public knowledgebase were completed by Molecule Annotation System 3.0 (MAS3.0). The Molecular Function and Biological progression of the differently expressed lncRNAs in urologic cancers were assessed by GO analysis, and the differently expressed lncRNAs related to biological pathways were detected by KEGG pathway analysis. *P* < 0.05 represented a significant difference.

### 2.4. Statistical Analysis

*T*-test or Mann–Whitney *U*-test was applied to perform statistical analysis. The survival function association was evaluated by the Kaplan-Meier curve method. One-way ANOVA was used for calculating the statistical significance among multiple groups. A significant statistical difference between or among comparison groups was shown as *P* < 0.05.

## 3. Results

### 3.1. Defining the Differently Expressed lncRNAs in Urologic Cancers

Here, the differently expressed lncRNAs in four sorts of urologic cancers, including PRAD, KIRC, KIRP, and BLCA, was identified by the lncRNAtor database [17]. Compared to normal samples, the differently expressed lncRNAs in cancer samples indicated that the gene expression should be ∣FC | >1.5 and *P* < 0.001. After comparison with normal samples, 297, 935, 602, and 287 lncRNAs were greatly dysregulated in BLCA, KIRC, KIRP, and PRAD samples, respectively, meaning lncRNAs exerted important function in urologic cancers. Hierarchical clustering showed the differently expressed lncRNAs in urologic cancers (Figures 1(a)–1(d)).

In comparison with the dysregulated lncRNAs in various cancer types, our data suggested that 34 lncRNAs were differently expressed in all four urologic cancer types. Among them, 18 lncRNAs (SNHG11, SNHG16, ZNFX1-AS1, GAS5, RPL32P3, AC005154.5, RP5-1180C10.2, SNHG1, ZNF761, PVT1, RP11-66N24.3, RP11-1149O23.3, TMEM191A, RP11-368I7.2, AP000525.8, AL589743.2, AL589743.1, and CTD-2314B22.3) were upregulated (Figure 1(e)) and 16 lncRNAs (MAGI2-AS3, SEMA3B, RP11-65F13.2, RP11-875O11.1, PLK1S1, LINC00476, RP11-57H14.4, RP5-842K24.2, MIR22HG, RP11-500G10.1, RP11-392A22.2, MED14-AS1, WDFY3-AS2, FGD5-AS1, RP4-669P10.18, and RPL23AP79) were downregulated (Figure 1(f)) in urologic cancers compared to normal tissues. Moreover, we identified cancer-type specific lncRNAs. We observed 37, 235, 105, and 132 lncRNAs were specifically upregulated in BLCA, KIRC, KIRP, and PRAD (Figure 1(e)), respectively. We also found 24, 187, 32, and 149 lncRNAs were specifically downregulated in BLCA, KIRC, KIRP, and PRAD (Figure 1(f)), respectively.

### 3.2. Construction of Common Differently Expressed lncRNAs Coexpressing Networks in Urologic Cancers

In this part, we conducted coexpression network analysis to forecast common differently expressed lncRNA functions in urologic cancers. In order to evaluate the correlation existing in differentially expressed mRNAs and lncRNAs, we selected lncRNA-mRNA pairs with ∣*R* | >0.7, and we established coexpression analysis. The Cytoscape software was applied then to construct coexpression networks. Coexpression network analysis demonstrated that 15 lncRNAs and 498 mRNAs were in KIRP and 5 lncRNAs and 386 mRNAs in KIRC, respectively (Figures 2(a) and 2(b)). Besides, the data illustrated that 14 lncRNAs and 1063 mRNAs were included in BCa, and 8 lncRNAs and 453 mRNAs were in PRAD (Figures 2(c) and 2(d)).

In view of our analysis, several lncRNAs were identified to be key regulators in the progression of urologic cancers. For example, MAGI2-AS3, PLK1S1, RP11-500G10.1, RP11-57H14.4, RP5-842K24.2, RP11-875O11.1, MED14-AS1, and RP11-65F13.2 in BLCA, RP5-1180C10.2, RP11-66N24.3, and FGD5-AS1 in KIRC, RPL32P3, RP11-66N24.3, RP5-1180C10.2, and SNHG11 in KIRC, and RP11-875O11.1, RP5-842K24.2, MAGI2-AS3, and FGD5-AS1 in PRAD were identified as key lncRNAs in coexpression networks.

### 3.3. Biological Functions of Common Differently Expressed lncRNAs Coexpressing Networks in Urologic Cancers

Then, we utilized the set of coexpressed mRNAs to analyze each lncRNA of the GO and KEGG pathway. We only displayed the top 10 lncRNAs closely related to the change of biological processes.  Figure 3 showed that the common differently expressed lncRNAs primarily participated in modulating histone deacetylation, RNA splicing, intracellular protein transport, regulation of mitophagy, and mRNA 3′-end processing in KIRC (Figure 3(a)) and also were involved in regulating translation, translational initiation, rRNA processing, proteasome-mediated ubiquitin, and DNA replication in KIRP (Figure 3(c)), in regulating muscle contraction, extracellular matrix organization, platelet aggregation, positive regulation of cell-substrate adhesion, and hippo signaling in PRAD (Figure 3(e)), and in regulating muscle contraction, extracellular matrix organization, positive modulation of GTPase activity, platelet degranulation, and negative modulation of transcription in BLCA (Figure 3(g)).

KEGG analysis showed that common differently expressed lncRNAs were enriched in biosynthesis of antibiotics, spliceosome, citrate cycle (TCA cycle), RNA transport, and carbon metabolism in KIRC (Figure 3(b)), ribosome, spliceosome, proteasome, Fanconi anemia pathway, and biosynthesis of amino acids in KIRP (Figure 3(d)), were associated with cGMP-PKG signaling pathway, focal adhesion, proteoglycans in cancer, actin cytoskeleton regulation, and vascular smooth muscle contraction in PRAD (Figure 3(f)), and were enriched in cGMP-PKG, oxytocin, MAPK, and calcium signaling pathways, dilated cardiomyopathy in BLCA (Figure 3(h)).

### 3.4. Construction of Cancer-Specific lncRNAs Coexpressing Networks in Urologic Cancers

We also constructed cancer-specific lncRNAs coexpressing networks in urologic cancers. Coexpression network analysis showed that 55 lncRNAs and 600 mRNAs were in PRAD, and 27 lncRNAs and 940 mRNAs were in BLCA, respectively (Figures 4(a) and 4(b)). Figures 4(c) and 4(d) indicated that 68 lncRNAs and 639 mRNAs were in KIRC, and 49 lncRNAs and 794 mRNAs were in KIRP.

According to our analysis, several cancer-specific lncRNAs were identified to be key regulators in the progression of urologic cancers. For example, LINC00607, PART1, AC025165.8, FAM138A, and RP11-175K6.1 in BLCA (Figure 5(a)), AC084018.1, HERC2P2, GOLGA2B, SH3BP5-AS1, CROCCP2, RP11-493K19.3, SEPT7P2, ZNF37BP, and RP11-228B15.4 in KIRC (Figure 5(b)), RP11-510M2.2, ZNF252P-AS1, UBE2Q2P2, ADORA2A-AS1, RP11-279F6.1, and MRPL23-AS1 in KIRP (Figure 5(c)), and RP1-163G9.1, LINC00675, AC003090.1, LINC00473, CYP4F8, AC017048.3, and ADAMTS9-AS1 in PRAD (Figure 4) were identified as key lncRNAs in cancer-specific lncRNAs coexpressing networks in urologic cancers.

### 3.5. Biological Functions of Cancer-Specific lncRNAs Coexpressing Networks in Urologic Cancers

Regarding cancer-specific lncRNAs, we conducted GO and KEGG pathway analyses. As shown in Figure 5, GO analysis revealed that KIRP-specific lncRNAs were mostly participated in morphogenesis of cilium, the process of metabolic, oxidation of fatty acid beta, homeostasis of lipid, and fatty acid beta-oxidation using acyl-CoA dehydrogenase (Figure 5(a)). PRAD-specific lncRNAs were main primarily taking part in modulating muscle contraction, transcription, extracellular matrix organization, cell-matrix adhesion, and cell migration (Figure 5(c)). BLCA-specific lncRNAs were mostly participated in modulating extracellular matrix organization, cell adhesion, angiogenesis, cell-matrix adhesion, and protein phosphorylation (Figure 5(e)). KIRC-specific lncRNAs were mainly taking part in the process of positive regulation of GTPase activity, T cell receptor signaling pathway, ubiquitin-dependent protein catabolic process, intracellular protein transport, and Golgi organization (Figure 5(g)).

KEGG analysis suggested that KIRP-specific lncRNAs principally took part in metabolic pathways, Staphylococcus aureus infection, biosynthesis of antibiotics, valine, leucine, and isoleucine degradation, and carbon metabolism (Figure 5(b)). PRAD-specific lncRNAs were enriched in focal adhesion, actin cytoskeleton regulation, vascular smooth muscle contraction, proteoglycans in carcinoma, and cGMP-PKG signaling pathway (Figure 5(d)). lncRNAs specific for BLCA were enriched in cGMP-PKG, oxytocin, MAPK, calcium, and cAMP signaling pathways (Figure 5(f)). KIRC-specific lncRNAs were enriched in T cell receptor, chemokine, Notch, TNF, and B cell receptor signaling pathways (Figure 5(h)).

### 3.6. Prognostic Implication of Differently Expressed lncRNAs in Urologic Cancers

GEPIA dataset was analyzed for further evaluating the assumed prognostic value of differently expressed lncRNAs in urologic cancers. Our data suggested that obvious relationships occur in these lncRNAs with the prognosis of cancer.

In the present study, we evaluate whether cancer-specific lncRNAs could serve as prognostic markers. We observed the dysregulation of TTC28-AS1 (Figure 6(a)) and RP11-613D13.8 (Figure 6(b)) in BLCA, the dysregulation of CTD-2006C1.2 (Figure 6(c)), NKAPP1 (Figure 6(d)), SDAD1P1 (Figure 6(e)), TP73-AS1 (Figure 6(f)), WWC2-AS2 (Figure 6(g)), SBF2-AS1 (Figure 6(h)), RP11-736K20.6 (Figure 6(i)), LINC00667 (Figure 6(j)), and ZNF826P (Figure 6(k)) in KIRC, the dysregulation of DLGAP1-AS3 (Figure 6(l)), SPON1 (Figure 6(m)), ULK4P3 (Figure 6(n)), RPL34-AS1 (Figure 6(o)), RP11-557H15.3 (Figure 6(p)), RP11-368J21.3 (Figure 6(q)), ANKRD18DP (Figure 6(r)), LINC00607 (Figure 6(s)), and ADORA2A-AS1 (Figure 6(t)) in KIRP, and the dysregulation of AC016700.5 (Figure 6(u)) and RP11-627G23.1 (Figure 6(v)) in PRAD were significantly correlated to overall survival time in urologic cancers.

Interestingly, we observed PVT1 was overexpressed in BLCA, KIRC, KIRP, and PRAD. Figures 6(w)–6(z) revealed that we found highly expressed PVT1 was negatively correlated with overall survival time in BLCA (Figure 6(w)), PRAD (Figure 6(x)), KIRC (Figure 6(y)), and KIRP (Figure 6(z)).

## 4. Discussion

Currently, urologic cancer mobility largely increased and it brought approximately 1,607,602 newly diagnosed cases worldwide, accounting for almost a quarter of the total number of human cancers in 2008. The commonly used biomarker for PCa diagnosis is the prostate-specific antigen (PSA) [18–20]. Unfortunately, there is not yet accurate and specific biomarkers for urologic cancer diagnosis or prognosis up to date, particularly for renal cell carcinoma and bladder cancer. lncRNAs belonging to noncoding RNA family and possessing the length of more than 200 bps were demonstrated to have an association with urologic cancer progression. For instance, Wan et al. observed androgen-responsive lncRNAs could serve as biomarkers for PCa [21]. PCA3 was observed to be more accurate than PSA in PCa detection [22–24]. Aggressive renal cell carcinoma was promoted by lncRNA MALAT1 via regulation of Ezh2 [25]. Here, we attempted to validate differently expressed lncRNAs in PRAD, BLCA, KIRC, and KIRP. Here, we found that 34 lncRNAs were differently expressed in all four urologic cancer types. Among them, 18 lncRNAs (SNHG11, SNHG16, ZNFX1-AS1, GAS5, RPL32P3, AC005154.5, RP5-1180C10.2, SNHG1, ZNF761, PVT1, RP11-66N24.3, RP11-1149O23.3, TMEM191A, RP11-368I7.2, AP000525.8, AL589743.2, AL589743.1, and CTD-2314B22.3) were upregulated and 16 lncRNAs (MAGI2-AS3, SEMA3B, RP11-65F13.2, RP11-875O11.1, PLK1S1, LINC00476, RP11-57H14.4, RP5-842K24.2, MIR22HG, RP11-500G10.1, RP11-392A22.2, MED14-AS1, WDFY3-AS2, FGD5-AS1, RP4-669P10.18, and RPL23AP79) were decreased in urologic cancers compared to normal tissues. Moreover, we identified cancer-type specific lncRNAs. We observed 37, 235, 105, and 132 lncRNAs were specifically increased and 24, 187, 32, and 149 lncRNAs were specifically upregulated in BLCA, KIRC, KIRP, and PRAD, respectively.

lncRNAs functioned crucially in the progression of human cancer via modulating cell proliferation, cisplatin resistance, migration, autophagy, and so on. lncRNAs could bind to DNA, proteins, and RNAs to influence target expression, translation, and activity. For instance, KCNQ1OT1 caused the alternation of tongue cancer proliferation and cisplatin resistance by modulating the miR-211-5p-mediated Ezrin/Fak/Src signaling pathway [26]. Nevertheless, the functions of most lncRNAs in human cancer needed further investigation. In our literature, coexpression analysis was performed to scoop out pivotal lncRNAs in urologic cancers. The roles of most of these lncRNAs were unclear. Only some lncRNAs, including MAGI2-AS3, PART1, LINC00675, and LINC00473 were reported to be linked with cancer growth. For instance, Chen et al. found LINC00473 expression was induced by CRTC1-MAML2 fusion and sustains human mucoepidermoid carcinoma cell growth and survival [27]. The long noncoding RNA LINC00473 contributes to cell proliferation via JAK-STAT3 signaling pathway by regulating miR-195-5p/SEPT2 axis in prostate cancer [28]. PART1 predicts a poor prognosis and promotes the malignant progression of pancreatic cancer by sponging miR-122 [29]. In NSCLC, lncRNA PART1 promotes cell proliferation and progression via sponging miR-17-5p [30]. Upregulation of LINC00675 as a ceRNA restrains hepatocellular carcinoma metastasis by sponging miR-942-5p [31]. In gastric cancer, LINC00675 suppresses cell proliferation and migration via downregulating the H3K4me2 level at the SPRY4 promoter [32]. The roles of differently expressed lncRNA were determined using GO and KEGG pathway analyses. We observed these differently expressed lncRNAs played crucial roles in urologic cancers via modulating muscle contraction, histone deacetylation, RNA splicing, translation, hippo signaling, etc.

TCGA database was analyzed to probe for the prognostic value of these dysregulated lncRNAs. Our data suggested that candidate lncRNAs had a great association with cancer progression. PVT1 was observed to be overexpressed in BLCA, KIRC, KIRP, and PRAD. Notably, our result revealed that highly expressed PVT1 represented a negative correlation with overall survival time in urologic cancers. In previous studies, ovarian carcinoma, pancreatic carcinoma, breast carcinoma, etc. highly expressed PVT1 [33–35]. Interestingly, previous studies had also demonstrated PVT1 was dysregulated in prostate, kidney, and bladder cancer [36, 37]. Mechanically, PVT1 could sponge miRNAs and bind proteins to modulate cell proliferation and invasion. For instance, He et al. reported that PVT1 mediated cell proliferation and invasion of colorectal carcinoma via stabilization of Lin28 and interaction with miR-128 [38]. In hepatocellular carcinoma, PVT1 promoted cell proliferation by recruiting Ezh2 [39]. These reports together with our analysis showed PVT1 could serve as a biomarker for human cancers. Moreover, we for the first time identified several cancers specifically expressed lncRNAs as biomarkers. For example, the dysregulation of RP11-613D13.8 in BLCA, the dysregulation of LINC00324 in KIRC, the dysregulation of RP11-557H15.3 in KIRP, and the dysregulation of LINC00668 in PRAD showed an obvious correlation with overall survival time in urologic cancers.

Several limitations should also be noted. For example, the conclusions in this study were obtained by analyzing TCGA database. In the future study, we will select clinical samples and detect the expression levels of these lncRNAs in cancer samples, which will further our findings. Secondly, loss of function assays should be performed to explore the potential biological functions of differently expressed lncRNAs in urologic cancers.

## 5. Conclusions

Our literature demonstrated comprehensively analyzed differently expressed lncRNAs in urologic cancers. Moreover, we performed bioinformatics analysis and found that differently expressed lncRNAs displayed multiple parts in different hormone-associated cancers. Additionally, our study gave prominence to the prognostic value of common and cancer-specific differently expressed lncRNAs in cancer outcomes, such as PVT1. Our research has deeply unearthed the mechanism of differently expressed lncRNAs in urologic cancer development.

## Figures and Tables

**Figure 1:** The differently expressed lncRNAs in urologic cancers. In the lncRNAtor database, 297, 935, 602, and 287 lncRNAs were identified to significantly dysregulated in (a) BLCA, (b) KIRC, (c) KIRP, and (d) PRAD. (e, f) The Venn diagram of the differently expressed lncRNAs in all four urologic cancers.

**Figure 2:** The common differently expressed lncRNAs coexpressing networks in urologic cancers. (a) The coexpression network of KIRP contains 14 lncRNAs and 498 mRNAs, (b) the coexpression network of KIRC contains 5 lncRNAs and 386 mRNAs, (c) the coexpression network of BLCA contains 14 lncRNAs and 1063 mRNAs, and (d) the coexpression network of PRAD contains 8 lncRNAs and 453 mRNAs.

**Figure 3:** Biological functions of common differently expressed lncRNAs coexpressing networks in urologic cancers. The GO and KEGG pathway analyses for common differently expressed lncRNAs coexpressing networks in (a, b) KIRC, (c, d) KIRP, (e, f) PRAD, and (g, h) BLCA.

**Figure 4:** The cancer-specific lncRNAs coexpressing networks in urologic cancers. (a) The coexpression network of PRAD contains 55 lncRNAs and 600 mRNAs, (b) the coexpression network of BLCA contains 27 lncRNAs and 940 mRNAs, (c) the coexpression network of KIRC contains 68 lncRNAs and 639 mRNAs, and (d) the coexpression network of KIRP contains 49 lncRNAs and 794 mRNAs.

**Figure 5:** Biological functions of cancer-specific lncRNAs coexpressing networks in urologic cancers. The GO and KEGG pathway analyses for cancer-specific lncRNAs coexpressing networks in (a, b) KIRP, (c, d) PRAD, (e, f) BLCA, and (g, h) KIRC.

**Figure 6:** Prognostic significance of differently expressed lncRNAs in urologic cancers. Several differently expressed lncRNAs were significantly correlated to overall survival time in (a, b) BLCA, (c–k) KIRC, (l–t) KIRP, and (u, v) PRAD. (w–z) PVT1 was significantly correlated to overall survival time in all four urologic cancers.

## Data Availability

Previously reported lncRNA data were used to support this study and are available at doi:10.1093/bioinformatics/btu325. These datasets are cited at relevant places within the text as references [17].
